The article "Analysis of Influencing Factors of College Students' Physical Exercise Habits Based on the Continuous Discrete Algorithm" was published in 2022. Journal: J Environ Public Health.

# Analysis of Influencing Factors of College Students' Physical Exercise Habits Based on the Continuous Discrete Algorithm

**DOI:** 10.1155/2022/2310438

**Published:** 2022-08-16

**Authors:** Zhijian Zhang, Miaomiao Jiang, Guanglong Shi, Shanshan Gao

**Affiliations:** ^1^School of Physical Education, South China University of Technology, Guangzhou 510006, China; ^2^Physical Education College of Harbin University of Commerce, Harbin 150028, China; ^3^Public Basic Institute, Anhui Medical College, Hefei 230601, China; ^4^Guangdong Technology College, Zhaoqing 526100, China

## Abstract

At present, college students give great importance to their physical training, but their physical habits are poor and they cannot exercise regularly. In view of the influencing factors in the habit formation of physical exercise, this paper puts forward a continuous discrete algorithm to provide students with a scientific and reasonable habit formation scheme. First, the data of college students' physical exercise habits are collected, and the data are cleaned and continuously analyzed to initially form a habit formation data set; Then, the information gain and clustering thought in the discrete algorithm are used to judge the data change, and the ordered relationship among the factors is obtained. Finally, in judging the influence degree of each factor, we find out the final influencing factors. MATLAB simulation shows that the continuous discrete algorithm can accurately analyze the problem of physical exercise habit formation and sort the influencing factors, with an accuracy rate of 90% and a calculation time of less than 19 minutes, which is significantly better than the original discrete algorithm.

## 1. Introduction

With the deepening of the reform of college students' physical education, colleges and universities pay more attention to the cultivation of exercise habits. However, there are many factors involved in the formation of physical exercise habits, and there are complicated relations among them, so it is necessary to comprehensively analyze the influencing factors. The cultivation of college students' physical exercise habits is a continuous process, which not only requires college students to persevere but also requires college students to constantly improve their exercise awareness and enhance their exercise self-confidence. College students' physical exercise habits are not only an important part of quality education but are also an inevitable requirement for college students to improve their physical quality. At present, the cultivation of college students' physical exercise habits lacksplanning and rationality, and even there are plans against the original intention of exercise, which is not conducive to the improvement of college students' physical health. Therefore, a comprehensive analysis of college students' physical exercise, combined with a variety of influencing factors and targeted exercise habits, has a very important theoretical and practical significance, in line with the current research trend. The key to improve college students' physical exercise habits is to analyze the influencing factors. The continuous discrete algorithm can not only analyze the relationship between influencing factors and the formation of physical exercise habits Xu et a. [1] but also mine the deep-seated structural relationship, which is the main method of intelligent data analysis at present. Literature research shows that discrete algorithms can classify data, eliminate irrelevant data, and improve the accuracy of data analysis Wu et al. [2]. However, in the process of data classification in discrete algorithms, external uncertainty will affect the analysis of factors and increase the error in the results. Some scholars also put forward a discrete analysis model, which can judge the influence degree between data Wang et al. [3], but the quantitative relationship between factors is relatively small. In the case of massive data, the discrete analysis model lacks comprehensive judgment ability, and the accuracy of the results will be greatly reduced Taheri et al. [4]. Therefore, some scholars put forward a continuous discrete algorithm to analyze the relationship between data and choose the corresponding progressive scheme Ognjenovic et al. [5], which can greatly improve the accuracy of the results and the research on this content shows an upward trend. The specific data are shown in Figure 1.

It can be seen from Figure 1 that the research on the cultivation of college students' physical exercise habits is increasing day by day, which shows that college students' physical exercise habits are the research hotspots in the future Liu et al. [6]. Freshmen's exercise plan is better than that of graduate students, their exercise evaluation is inferior to that of graduate students, and there is no difference in exercise habits between freshmen and graduate students. The crossresults between the influencing factors of physical exercise and the cultivation conditions are shown in Table 1.

It can be seen from Table 1 that the crosscoefficients between the influencing factors and the habit formation conditions are all greater than 0.3, indicating that there is an inevitable correlation between the influencing factors and the habit formation conditions, and the latter influencing factors can be analyzed. At the same time, it is found that the frequency of exercise habits and the systematicness of exercise are the main factors, which are beneficial to the cultivation of college students' physical exercise habits. In addition, exercise awareness is also a key factor to develop exercise habits, so we should help college students develop exercise habits from the perspective of the abovementioned factors. The advantage of a continuous discrete algorithm lies in the large amount of data processing, continuous analysis of problems, and more comprehensive and specific analysis results, which are suitable for dealing with complex problems. Physical exercise habits are continuous problems. The continuous discrete algorithm can explore the problems in the cultivation of exercise habits, and by comparing the results of different periods, the problems can be deeply excavated and the analysis results are more accurate. Compared with the continuous discrete algorithm, traditional ant colony, regression, Bayesian, and other methods have a single analysis process and simple data processing, which cannot realize continuous analysis. At present, there are many research studies on the continuous discrete algorithm in foreign countries, but there are relatively few research studies in China, and there are fewer research studies on physical exercise learning. Therefore, the research of this paper is of great significance.

## 2. Concepts Related to the Continuous Discrete Algorithm

### 2.1. Mathematical Description of the Formation of College Students' Physical Exercise Habits

The continuous discrete algorithm is a continuous algorithm based on distance and information gain. The basic idea of this algorithm is clustering and information gain. The continuous discrete algorithm can not only analyze the relationship between attributes and values of data and form an orderly analysis result but also judge the value of attributes. A continuous discrete algorithm has obvious advantages, mainly reflected in continuity analysis, which can judge data more accurately. Discrete data meet the actual analysis requirements and can be used for data attribute analysis. In addition, the continuous discrete model can reduce the amount of continuous data analysis, better describe the data, improve the calculation speed, and reduce the occupation of redundant data to system resources. Compared with other algorithms, the continuous discrete algorithm can automatically adjust the threshold, meet the requirements of analysis results, and improve the consistency of results. In order to further analyze the problem, it is necessary to describe the problem mathematically as follows.

**Hypothesis 1 .**

.The data sample of college students' physical exercise habit formation *X*=(*x*_*i*_, *y*_*i*_*|*_*t*_), the influencing factors are*d*_*i*_, and the influence degree of each factor on habit formation is *q*_*i*_; then, the physical exercise habit formation function is *F*(*d*_*i*_, *q*_*i*_, *b*_*i*_, *X*)_*t*_. The values in the function *F*(*d*_*i*_, *q*_*i*_, *b*_*i*_, *X*)_*t*_ correspond to unique results, and the results are mapped into plane space$S\left(X_{i},{\overset{⟶}{X}}_{i}\right)$ where *X*_*i*_ is the mapping value and ${\overset{⟶}{X}}_{i}$ is the mapping attribute [5]. The mapping distance between the values is, and the values represent the accuracy of the analysis results. The specific calculation process is shown in formula (1).

(1) $$\begin{array}{c} S=w\cdot S\left(X_{i},{\overset{⟶}{X}}_{i}\right)+\lambda \cdot F{\left(d_{i},q_{i},b_{i},X\right)}_{t}, \end{array}$$

where *w* is the threshold of mapping and *λ* is the weight body of the function. At *S* < 0, the influence of representative influencing factors was negative [6], and at *S* > 0, the influence of representative influencing factors was positive.

**Hypothesis 2 .**

.If the time of physical exercise habit formation is continuous *T*_*i*_ ∈ [0,1], it shows that the data samples are continuously discrete and mapped to the threshold *w* > 0.5. Then, the calculation of _*S*_ is as shown in formula (2).

(2) $$\begin{array}{c} S=w\cdot \lambda \cdot \sum T_{i}\cdot F\left(d_{i},q_{i},b_{i},X\right). \end{array}$$

**Assumption 1 .**

.If *F*(*d*_*i*_, *q*_*i*_, *b*_*i*_, *X*) < (2*d*_*i*_+4*q*_*i*_ · *b*_*i*_+*X*^2^/2*d*_*i*_ · *q*_*i*_ · *b*_*i*_) is a function, it is as shown in formula (3).

(3) $$\begin{array}{c} S\left(X_{i},{\overset{⟶}{X}}_{i}\right)=\sin\;\theta_{i}\cdot F\left(d_{i},q_{i},b_{i},X\right)|t. \end{array}$$

Among them, ${\overset{⟶}{X}}_{i}$ is the vector of *X*_*i*_, *θ* is the angle between influencing factors and mapping points, and *t* reflects the time continuity of influence in space. The influencing factors are *d*_*i*_, the influence degree of each factor on habit formation is *q*_*i*_; then, the physical exercise habit formation function is *F*(*d*_*i*_, *q*_*i*_, *b*_*i*_, *X*)_*t*_. Therefore, the *θ* and *t* in the continuous discrete method are the keys to judge the influence of factors on the results as shown in Figure 2.

As can be seen from Figure 2, continuous data can be standardized to obtain two-dimensional projection results. After angle analysis, regular data sets can be obtained from irregular data. Irregular data represent the random data of college students' physical exercise. After standardized processing, regular data can be obtained, which can be better analyzed. Therefore, continuous discrete analysis can standardize the rule data and meet the continuous analysis of college students' exercise habits, which has strong advantages.

According to Figure 2, the discreteness of data is analyzed and the result is shown in Figure 3.

According to Figure 3, it can be seen that the relationship between the data of college students' physical exercise habits and time and angle is discrete, and the data are equidistant. This shows that there is no correlation between the data, which meets the requirements for continuous discrete analysis of data and can be used for subsequent analysis.

### 2.2. Continuous Discrete Algorithm

The single discrete algorithm mainly simulates exercise habits, including personal interests, exercise habits, imitating others, and realizing data analysis of physical exercise habits. At the early stage of habit formation, the number of physical exercise and physical exercise habits is the same Li et al. [7]. Different physical exercises are affected by different factors. We randomly obtain the data of college students' physical exercise habits, select the influencing factors with higher influence degree, analyze the influence degree with this influencing factor as the core, and reduce 1/2 of the influencing factors by sorting the influencing factors. Then, the factors that have the most obvious influence on habit formation are selected by iterative calculation, and the corresponding weights are given Guedes et al. [8].

Assuming that the discrete initial number of influencing factors is *n*, and the random influence degree of influencing factors is $S\left(X_{i},{\overset{⟶}{X}}_{i}\right)$, *x*_*i*_, *y*_*i*_ is the complexity and depth of physical exercise, and *z*_*i*_ is the influencing factors of different habit formation; then, the discrete initial influence degree of physical exercise habit formation is as shown in formula (4).

(4) $$\begin{array}{c} S\left(X_{i},{\overset{⟶}{X}}_{i}\right)=\frac{w\cdot \lambda \cdot F\left(d_{i},q_{i},b_{i},X\right)}{T_{i}}. \end{array}$$

Among them, the random influencing factors of physical exercise habit formation of college students are *x*_*i*_, *y*_*i*_, and*z*_*i*_; *T*_*i*_ is the continuous values of influencing factors. We randomly select the influencing factors, cross-judge, and iterate the influence degree of the influencing factors. Under the constraint of exercise standard, we judge the influence degree of factors as shown in formula (5).

(5) $$\begin{array}{c} S\left(X_{i},{\overset{⟶}{X}}_{i}\right)=w\cdot \sum F\left(d_{i},q_{i},b_{i},X\right)⟶\sum \lambda F\left(d_{i},q_{i},b_{i},X|T\right). \end{array}$$

Among them, *i* ∈ [0, *n*/2].

The influence of factors on exercise habits is *p*_*i*_ based on discrete probability. Whether each factor has normality is judged by discrete probability calculation, and the neighborhood judgment of the influencing factors with normality is carried out to obtain the corresponding discrete probability S. Golia [9]. The judgment process is as shown in formula (6).

(6) $$\begin{array}{c} p_{i}=\frac{F\left(d_{i},q_{i},b_{i},X\right)}{\sum_{i}^{n}\left[R\left(x,y\right)|T\right]}. \end{array}$$

Among them, *R*() is the discreteness of influencing factors.

If the best value of college students' physical exercise habits is still not obtained after iterative calculation, the search for this influencing factor will be abandoned and other influencing factors will be analyzed Fan et al. [10]. At the same time, according to formula (4), new influencing factors are randomly obtained here for the next judgment.

The adjustment of impact degree. In the initial stage of dispersion, if the judgment of influence degree cannot guarantee the comprehensiveness, the overall performance of the judgment result of influence degree will be reduced Xu et al. [11]. Therefore, in the process of influencing factor analysis, we should try our best to expand the judgment range, narrow the judgment range near the main influencing factors of habit formation, and constantly adjust the factors to improve the success rate of habit formation. Assuming that the adjustment rate is set to the degree of judgment factor, the recognition rate of the main influencing factors is calculated as shown in formula (7).

(7) $$\begin{array}{c} \phi =\sum \Delta \nu_{i}R\left(x,y\right). \end{array}$$

Among them, Δ*ν*_*i*_ is the change of influence degree.

Among them, it is the change of influence degree.

(8) $$\begin{array}{c} \Delta {}_{L}\left(x_{i},y_{i},z_{i}\right)=w\cdot F\left(d_{i},q_{i},b_{i},X\right)+\lambda \cdot \nu_{i}\cdot S\left(X_{i},{\overset{⟶}{X}}_{i}\right). \end{array}$$

From formula (7), it can be seen that the value *F*(*d*_*i*_, *q*_*i*_, *b*_*i*_, *X*) is relatively small and *ν* is large in the initial stage of dispersion, so it is necessary to continuously expand the data collection Mews et al. [12] and keep the comprehensiveness of the influencing factor analysis. In the later stage of discretization, the values *F*(*d*_*i*_, *q*_*i*_, *b*_*i*_, *X*) is relatively large and *ν* is relatively small, so it is necessary to continuously mine numbers to improve the analysis depth of continuous discrete algorithm. The specific results are shown in Table 2.

The mining depth, scope, and sample number of influencing factors of refining all meet the actual requirements. This shows that the adjustment of data samples of college students' physical exercise habits meets the requirements of data analysis and can be used for later data analysis.

The introduction of iteration factor. When a certain influencing factor is comprehensively analyzed many times and reaches the analysis limit, personal interest will be changed into the deep excavation, looking for new influencing factors, and judging new influencing factors Kuzmin et al. [13]. Due to the strong randomness and poor antidisturbance ability of college students influence degree judgment, errors will appear in the early stage of influence degree analysis. In order to reduce the occurrence probability of errors in the formation of college students' physical exercise habits, this paper introduces adjustment factors, reduces the uncertainty of physical exercise through probability density function, and helps college students to reduce errors in the formation of physical exercise habits. The calculation formula of adjustment factors is as shown in formula (9).

(9) $$\begin{array}{c} S\left(X_{i},{\overset{⟶}{X}}_{i}\right)=\sin\;\theta \cdot F\left(d_{i},q_{i},b_{i},X\right). \end{array}$$

When *F*(*d*_*i*_, *q*_*i*_, *b*_*i*_, *X*) is 1, *F*(*x*_*i*_, *y*_*i*_, *z*_*i*_) can be expressed by the adjustment factor distribution function Cauthy (0, 1). When *F*(*d*_*i*_, *q*_*i*_, *b*_*i*_, *X*) is 0, the external uncertainty of physical exercise is the highest; otherwise, the uncertainty is the lowest Gao et al. [14]. Because the two sides of Cauthy (0, 1) tend to an extreme value slowly, its distribution speed is less than Gauss (0, 1), thus reducing the uncertainty of physical exercise. Moreover, the peak value of Cauthy (0, 1) is smaller than that of Gauss (0, 1), which weakens the influence of other factors. Based on the above analysis, the judgment formula of physical exercise adjustment factors can be transformed into formula (10).

(10) $$\begin{array}{c} \Delta S{\left(X_{i},{\overset{⟶}{X}}_{i}\right)}_{t}=F\left(d_{i},q_{i},b_{i},X\right)*t. \end{array}$$

### 2.3. Analysis of the Habit Formation Scheme

The rationality of the habit formation scheme is the main factor to measure the continuous discrete algorithm. An analysis of the influence degree of college students on personal interests, exercise habits, and other operations Ennaji et al. [15] can not only measure the relationship between physical exercise and physical exercise habit formation and perfection but also improve the accuracy of habit formation and perfection. From formula (8), we can see that when judging the influencing factors of physical exercise in the initial stage, we pay great attention to the analysis of comprehensive factors, and when judging the influencing factors in the later stage, we pay attention to the cultivation and perfection of physical exercise habits. At the same time, according to different physical exercise habits, we choose different habit formation schemes. At present, besides the continuous discrete algorithm, there are other improved habit formation schemes .

(1) personalize the scheme as shown in formula (11).
  (11) $$\begin{array}{c} \Delta S\left(X_{i},{\overset{⟶}{X}}_{i}\right)=S\left(X_{i},{\overset{⟶}{X}}_{i}\right)\cdot p_{i}. \end{array}$$
The specific iterative process is shown in Figure 4.
As can be seen from Figure 4, there is a linear relationship between personalized schemes and time, and there is no correlation between various schemes, which shows that the whole analysis result is independent and later operations can be carried out. In addition, the individuation rate of the scheme is 60%, slightly higher than 50%, so the individuation of the overall scheme is strong, which can meet the physical exercise requirements of college students.
(2) comprehensive scheme is as shown in formula (12).
  (12) $$\begin{array}{c} \Delta S\left(X_{i},{\overset{⟶}{X}}_{i}\right)=F\left(d_{i},q_{i},b_{i},X\right)-R\left(x,y\right). \end{array}$$
The specific analysis process is shown in Figure 5.
(3) scheme success rate is as shown in formula (13).
  (13) $$\begin{array}{c} \Delta S\left(X_{i},{\overset{⟶}{X}}_{i}\right)=\tan\;\theta ÷\sum_{i=1,t}^{n/2}\Delta L_{i-1}\left(o\right). \end{array}$$
The specific analysis process is shown in Figure 6.
(4) multifactor scheme is as shown in formula (14)
  (14) $$\begin{array}{c} \Delta S\left(X_{i},{\overset{⟶}{X}}_{i}\right)=\sum_{t}\Delta S\left(X_{i},{\overset{⟶}{X}}_{i}\right)÷n \end{array}$$
The specific analysis process is shown in Figure 7.

Among them, *T* is the time for college students to develop their physical exercise habits.

In this paper, the continuous discrete algorithm is improved in two aspects: on the one hand, mapping weight *w* and mapping threshold *λ* are set every time the influence degree is analyzed by Colbrook [16]. At the same time, the continuous discrete algorithm randomly selects five habit formation schemes and completes many improvements in physical exercise habit formation. In the later stage of influence degree judgment, the judgment space is gradually reduced, neighborhood judgment is carried out, and the diversity of influence degree judgment of college students is maintained to improve the comprehensiveness of judgment. On the other hand, balancing the relationship between different influencing factors and incorporating iterative factors Δ*ν*_*i*_*r*Δ*ν*_*i*_, moderate function *F*(*x*_*i*_, *y*_*i*_, *z*_*i*_), and Lagrangian multiplier function can judge the formation of performance habits more accurately.

Data analysis on the synergistic effect of different college students' physical exercise influencing factors. Collaborative analysis of influencing factors is the main way to improve the physical exercise habit formation scheme. Based on the analysis of influencing factors of college students' physical exercise, this model constructs a discrete habit formation data set Aristodimou et al. [17]. Different subsets adopt different collaborative schemes, influencing factors, and collaborative operations. The influencing factors are randomly divided into five subsets, and each subset represents a subspace. In each iteration, the subset will randomly choose different collaborative analysis strategies. Every physical exercise habit will be comprehensively analyzed. After completion, we compare the influence degree of different subsets and the complexity of the physical exercise and record the best habit formation; Other subsets are aggregated to the best habit formation scheme to improve the judgment efficiency of influencing factors.

### 2.4. Steps of Developing College Students' Physical Exercise Habits Based on the Continuous Discrete Algorithm

The basic idea of the continuous discrete algorithm is to use a variety of collaborative methods to optimize the threshold and weight in the habit formation scheme Alsadat et al. [18], obtain the main influencing factors of physical exercise, and improve the habit formation of physical exercise. The implementation steps of this model are shown in Figure 2:

  Step 1: Determine the structure and uncertainty of physical exercise. According to the characteristics of practical problems, determine the nonlinear distribution structure of physical exercise, as well as the uncertainty, the uncertainty of college students' physical exercise habits.
  Step 2: Habit formation initial physical exercise habit formation. According to the relevant factors, college students' physical exercise habits are formed in the initial stage. The number of college students' physical exercise habits is *n* = 30, the number of physical exercises is consistent with that of college students' physical exercise habits, and the iterative times are *m* = 50.
  Step 3: Determine the fitness function. Using discrete theory, the influencing factors of college students' physical exercise are randomly obtained, and they are mapped to plane space, and the mapping vector weight and mapping threshold at the initial stage of discrete are obtained. According to the requirements of physical exercise habits, the weights and thresholds are set. Through formulas (3)∼(7), the influence of each factor on college students' physical exercise habits is analyzed.
  Step 4: Judge the physical exercise habit formation plan. The influencing factors at the initial stage of discretization are divided into five subsets; the fitness is obtained, and the best scheme and the main factors of subinfluencing factors are compared.
  Step 5: Iteration of influencing factors. We adjust the adjustment factor, randomly select the analysis strategy from five schemes, and calculate according to formula (2) and formula (7).
  Step 6: Collaborative analysis of influencing factors. After an influencing factor analysis, we select the main influencing factors, obtain the corresponding cultivation program, carry out other influencing factors analysis, carry out influence degree analysis, and get the final influencing factor list.
  Step 7: Judge whether the influencing factor reaches the maximum value *m* and whether the iteration times reach *m*. If it has been reached, we repeat steps 1∼5, otherwise stop the analysis of influence degree and return to threshold, weight, and best habit formation scheme.

## 3. Empirical Analysis

### 3.1. Analysis of Judgment Results

In order to further verify the judgment results of the continuous discrete algorithm, this paper analyzes from four angles: interest, consciousness, conformity, and fitness, and constructs corresponding functions. The specific process is as follows .

(1) Interest function, and the result is shown in formula (15)
  (15) $$\begin{array}{c} A\left(x\right)=\sum_{i=1}\frac{x_{i}^{2}}{n}+p_{i}. \end{array}$$
The specific iterative process is shown in Figure 8
As can be seen from Figure 8, the dispersion of interest function is high, which meets the analysis requirements
(2) Consciousness function, the result is shown in formula (16)
  (16) $$\begin{array}{c} B\left(x\right)=\sum_{i=1}\sqrt{p\cdot x_{i}^{2}}. \end{array}$$
(3) Conformity function, the result is shown in formula (17)
  (17) $$\begin{array}{c} C\left(x\right)=\frac{e}{20}+\left|e^{p}\right|. \end{array}$$
(4) Fitness function, the result is shown in formula (18)
  (18) $$\begin{array}{c} D\left(x\right)=p+\sum_{i=1}\frac{x_{i}^{2}}{n}, \end{array}$$
where I is 1 and 2. We obtain the minimum value 0, at (0, 1). Related parameter settings: The total number of influencing factors is 20, the number of iterations is 100, and each group of experiments is carried out independently. The test results are shown in Table 3.

As can be seen from Table 3, the continuous discrete algorithm is superior to the single discrete algorithm, with a higher matching degree and more theoretical best schemes. In terms of interest and awareness, the accuracy of the continuous discrete model is more than 90%, the average accuracy is more than 80%, the standard deviation is less than 0.23, and the influence degree is more than 80%, which is superior to the discrete method. Therefore, the calculation results of the continuous discrete analysis method are better. Moreover, the value range, average value, and judgment error of a continuous discrete algorithm are smaller than those of a single discrete algorithm. In order to verify the performance of the continuous discrete algorithm more intuitively and judge the perfection of this technology in the cultivation of physical exercise habits, the following analysis graphs are given. See Figure 9.

As can be seen from Figure 9, the interest shows irregular changes and changes to the degree of concentration, which shows that the convergence of the interest function is better.

As can be seen from Figure 10, the change of the consciousness function is more concentrated and more concentrated.

As can be seen from Figure 9–11, the continuous discrete algorithm is faster and more stable, which is superior to the single discrete algorithm. Therefore, the continuous discrete algorithm has better performance in judgment speed and judgment accuracy, and the judicial process is more stable, which is suitable for multifactor analysis.

### 3.2. Data Processing of Physical Exercise Habit Formation

In this paper, 12 universities were selected as research objects, and 1023 influencing factor data were collected as research data samples, which were collected from January 1, 2022, to June 12, 2022. After preliminary screening and sorting of influencing factors, 872 data of influencing factors were obtained. According to the physical exercise standards stipulated by the state, the influencing factors are classified into four categories, namely, the main influencing factors, the secondary influencing factors, the subjective influencing factors, and the objective influencing factors. The results are shown in Table 4. This paper judges the accuracy of the results according to theoretical judgment and practical verification.

### 3.3. The Results of Developing College Students' Physical Exercise Habits

According to the experimental situation, we determine the results of college students' physical exercise habits. In this paper, a continuous discrete algorithm is proposed to classify the influencing factors, and the corresponding results are obtained as shown in Figure 12.

As can be seen from Figure 12, the data sample classification of the continuous discrete algorithm is discrete, which is closer to the actual data distribution, while the single discrete algorithm concentrates on the classification of influencing factors, which cannot meet the analysis needs of college students' physical exercise habit formation scheme. In addition, the data sample distribution of a continuous discrete algorithm is not affected by external factors, while the data sample distribution of a single discrete algorithm is affected by uncertainty and is more concentrated. The reason is that the continuous discrete algorithm incorporates adjustment coefficients and thresholds, maps influencing factors to plane space, and realizes standardized processing of factor data. Comparing the evaluation effects of different methods on college students' physical exercise habits, they are mainly: single discrete algorithm, statistical algorithm, continuous discrete algorithm, and questionnaire. The results are shown in Figure 13.

As can be seen from the above figure, the continuous discrete algorithm has the highest influence and reaches the limit at the earliest. Under the same uncertainty, the stability of the continuous discrete algorithm is higher, followed by single discrete algorithm, statistical algorithm, and questionnaire. The reason is that the continuous discrete algorithm reduces the influence of uncertainty on the judgment results, and the continuous discrete algorithm provides different habit formation schemes to improve the accuracy of physical exercise habit formation and improvement results, which is consistent with relevant research. From the main influencing factors, this paper analyzes the accuracy of different techniques in developing physical exercise habits and the results are shown in Table 5.

As can be seen from the above table, the success rate of physical exercise habit formation based on the continuous discrete algorithm is high, and the accuracy rate does not change with the types of influencing factors. The main reason is that the adjustment factor's analysis of data samples makes its continuous judgment time shorter and can make the change of habit formation scheme more flexible. Therefore, the continuous discrete algorithm can not only reduce the influence of factors on habit formation but also improve the success rate of physical exercise habit formation.

## 4. Conclusion

Based on the discrete theory and the continuous discrete method of continuous analysis, this paper analyzes the influencing factors of college students' physical exercise habits. By setting threshold, weight, and the synergy method, we find out the main influencing factors and help college students choose a reasonable habit formation scheme. The continuous discrete algorithm can classify data samples discretely, make the distribution of data samples closer to the actual distribution, and improve the accuracy of analysis results. MATLAB simulation results show that the continuous discrete algorithm, which found the main influencing factors, mining the deep content of habit formation, has a higher success rate in college students' physical exercise habit formation. In terms of interest, consciousness, and habit, the accuracy of the continuous discrete model is more than 90%, the average accuracy is more than 80%, the standard deviation is less than 0.23, and the influence degree is more than 80%, which is significantly superior to the discrete method and can be used as a guiding method for college students to develop physical exercise habits. However, there are still some shortcomings in the switching of different influencing factors. In the future, we will focus on the transition between different factors to improve the effectiveness of the continuous discrete algorithm.

## Figures and Tables

**Figure 1:** Research on the formation of college students' physical exercise habits in 2021.

**Figure 2:** Spatial projection of influencing factors.

**Figure 3:** Discrete analysis of angle and time data.

**Figure 4:** Iterative relationship between personalization scheme and time.

**Figure 5:** Iterative relationship between comprehensive scheme and time.

**Figure 6:** Iterative relationship between success rate and time.

**Figure 7:** Iterative relationship between multi-factors and time.

**Figure 8:** Analysis process of interest function.

**Figure 9:** Analysis curve of influence degree of the interest function.

**Figure 10:** Analysis curve of influence degree of the consciousness function.

**Figure 11:** Analysis curve of influence degree of the conformity function.

**Figure 12:** Discrete results of data samples.

**Figure 13:** Comparison of influence degree of different methods.

**Table 1:** The crossresults between influencing factors and habit formation conditions.

	Fun	Motivation	Health	Socialize	System	Obedience	Appearance
Exercise time	0.55	0.42	0.56	0.44	0.45	0.17	0.17
Exercise intensity	0.59	0.44	0.40	0.51	0.29	0.45	0.21
Exercise frequency	0.61	0.46	0.68	0.64	0.50	0.18	0.64
Habit formation	0.45	0.58	0.59	0.68	0.67	0.60	0.14
Exercise consciousness	0.66	0.58	0.45	0.61	0.18	0.65	0.54

(Source: CNKI, Wanfang and Weipu).

**Table 2:** Analysis criteria of influencing factors of habit formation in different stages.

Stage	Indicators	Number of samples	Excavation depth	Range expansion rate	Number of characteristic solutions
Prestage	Fun	47^*∗*^	36.26	29.86	3
	Motivation	58	51.18	29.86	5
	Health	15	46.92	93.84	6
	Socialize	42	42.65	49.05	6
	System	27	81.04	42.65	5
	Obedience	59	34.12	44.79	6
	Obedience	31	74.64	95.97	1
Later stage	Fun	20^*∗*^	61.85	63.98	3
	Motivation	23^*∗*^	31.99	36.26	5
	Health	23^*∗*^	42.65	57.58	1
	Socialize	36^*∗*^	89.57	83.17	1
	System	31^*∗*^	46.92	70.38	2
	Obedience	47^*∗*^	72.51	42.65	3
	Obedience	62^*∗*^	68.24	46.92	2

Compared with the previous period, ^*∗*^*P* < 0.05.

**Table 3:** The judgment results of each index.

Function	Method	Accuracy	Calculating time	Average accuracy	Standard deviation	Degree of influence	Nurturing rate
Interest	Continuous discretization algorithm	86.50	4	77.75	0.37	68.24	81.64
	Discretization algorithm	89.42	11	79.70	0.30	89.57	83.58
Consciousness	Continuous discretization algorithm	91.36	19	81.64	0.23	81.04	86.50
	Discretization algorithm	92.33	6	88.44	0.32	81.04	91.36
Conformity	Continuous discretization algorithm	79.70	11	91.36	0.20	31.99	90.39
	Discretization algorithm	89.42	20	90.39	0.15	38.39	78.72

Data source: Questionnaire, interview outline.

**Table 4:** Collection of the number and proportion of influencing factors.

Classification of influencing factors	Number of factors (pieces)	Degree of influence
Main influencing factors	43	92.1
Secondary influencing factors	31	95.15
Subjective influencing factors	23	91.23
Objective influencing factors	98	90.42

**Table 5:** The success rate of different methods to develop physical exercise habits.

Classification of influencing factors	Continuous discrete algorithm	Single discrete algorithm	Statistical algorithm	Questionnaire
Main influencing factors	99.34	98.33	97.32	96.31
Secondary influencing factors	99.31	95.34	95.33	92.31
*T*	5.83	14.58	12.63	10.20
*P*	0.00	0.02	0.01	0.01
Subjective influencing factors	99.31	95.34	95.33	92.31
Secondary influencing factors	99.37	98.32	98.37	98.30
*T*	9.72	7.78	8.97	12.63
*P*	0.01	0.01	0.01	0.02
Objective influencing factors	99.34	97.32	94.33	95.36
Main influencing factors	99.34	98.33	97.32	96.31
*T*	0.97	1.94	0.97	5.83
*P*	0.00	0.01	0.01	0.02
Objective influencing factors	99.34	98.33	97.32	96.31
Subjective influencing factors	99.31	95.34	95.33	92.31
*T*	3.89	3.89	6.80	12.63
*P*	0.01	0.02	0.01	0.03

## Data Availability

The data used to support the findings of this study are available from the corresponding author upon request.
